# A Novel Keyword Generation Model Based on Topic-Aware and Title-Guide

**DOI:** 10.1155/2022/1787369

**Published:** 2022-05-23

**Authors:** Jialin Ma, Jieyi Cheng, Yue Zhang

**Affiliations:** College of Computer Science, Huaiyin Institute of Technology, Huaian 223003, China

## Abstract

Keywords are usually one or more words or phrases that describe the subject information of the document. The traditional automatic keywords extraction methods cannot obtain the keywords which do not appear in the document, and the semantic information is not considered in the extraction process. In this paper, we introduce a novel Keyword Generation Model based on Topic-aware and Title-guide (KGM-TT). In the KGM-TT, the neural topic model is used to identify the latent topic words, and a hierarchical encoder technology with attention mechanism is able to encode the title and its content, respectively. The keywords are generated by the recurrent neural network with attention and replication mechanism in our model. This model can not only generate the keywords which do not appeared in the source document but also use the topic information and the highly summative word meaning in the title to assist the generation of keywords. The experimental results show that the *F*1 value of this model is about 10% higher than that of CopyRNN and CopyCNN.

## 1. Introduction

Keyword is the smallest unit to express the subject meaning of a document. It is widely used in tasks such as information retrieval, documents classification, and opinion mining [1]. With the rapid development of the Internet, the number of electronic documents is increasing exponentially. Various methods of automatically extracting and generating keywords have been proposed. The main step of traditional automatic keyword extraction methods (such as n-gram, TF-IDF, TextRank [2], SingleRank [3], and KEA [4]) is to identify candidate words and then rank all the candidates based on the importance computed by either unsupervised ranking approaches or supervised machine-learning approaches [5]. The keywords extracted by the above methods are words that have appeared in the source file, such as the keywords “knowledge graph,” “knowledge resolution,” and “relation embedding” in Figure 1. However, according to relevant research statistics, nearly half of the keywords given by the author in the scientific articles do not appeared in the source document [6], such as the keywords “knowledge representation” and “entity embedding” in Figure 1. Therefore, these kinds of extracting methods cannot generate keywords that do not appear in the source document, and they are difficult to mine the deep semantic information between context words.

To overcome the above drawbacks, some researchers had proposed a Sequence-to-Sequence model to solve the keyword generation task and had achieved some results, including seq2seq, CopyRNN [6], CorrRNN [7], and CopyCNN [8]. First, these methods treat the title and the main body content equally and just combine them as the source document input. Then, the encoder is used to maps each document word to a hidden state vector as the context representation. Finally, a decoder based on context representation is used to generate keywords from a predefined vocabulary [9]. However, these generation methods still have some flaws. They do not consider whether keywords exist in the document but directly extract them from the vocabulary, so they can generate keywords that do not appear in the source document. In fact, the title is the core subject condensed by the document author. However, they ignore the guiding role of title on keyword generation and fail to give full play to the strong semantic information of document title.

The title is a highly purified and refined for the document, which can accurately reflect the nature, scope, and depth of the content of the document. Keywords are words that can express the characteristics of document subject content, and they play a similar and complementary role with title [10], so keywords and titles have similar semantic information. Taking an academic paper as an example, the title is usually straightforward, focused, concise, and directly expounds the research object, research method, and research purpose of the paper. Therefore, one or several main central words in the title can often be directly used as keywords [4]. As shown in Figure 1, “relation embedding” in keywords appears in the title but not in the body. In addition, the information in the title also helps to reflect which parts of the body of the document are important, such as including the same or related parts as the title.

In view of the fact that the existing extractive methods does not fully consider the semantics of context and the generative models ignore the guiding role of title, in this paper, we propose a Keyword Generation Model based on combination Topic-aware and Title-guide (KGM-TT). First, the neural topic model based on the variational autoencoder is used to generate the latent topic of the document and the hierarchical encoder with attention mechanism to encode the corpus; then, the circular neural network with attention copy mechanisms to decode the corpus coding and topic distribution for generating keywords. The KGM-TT model not only enriches semantic features by mining latent topics but also uses highly summative and valuable information in the title to jointly guide the generation of keywords.

## 2. Related Works

### 2.1. Keyword Extraction

At present, there are many keyword extraction methods, which are mainly divided into unsupervised methods and supervised methods [5]. For unsupervised extraction methods, Mihalcea and Tarau [2] proposed the TextRank-based graph ranking method to calculate the correlation between candidate keywords. Liu et al. [11] used the KeyCluster method of clustering to detect representative phrases from topic clusters. For supervised machine learning methods, the keyword extraction task is transformed into a binary classification problem [7]. Firoozeh et al. [4] introduced KEA method, which extracts candidate phrases from documents, then calculates several features such as TF-IDF value and location information of each candidate phrase, finally they used Naive Bayes model (NB) to judge whether the candidate words are keywords. Turney [12] adopted C4.5 decision tree training classifier. Wang and Peng [13] used Support Vector Machine (SVM) to extract keyword usage features, including word frequency and location information of words. Zhang [14] used Conditional Random Field (CRF) to extract keywords from documents.

The above extraction methods still cannot generate keywords that are not in the source documents. With the development of deep learning technology, a growing number of researches have been gradually evolving from keyword extraction to generative method [5]. Liu et al. [15] proposed to view the keywords extraction task from the perspective of machine translation. They modeled the keywords extraction process as a translation operation from document to keywords and took the keywords as the target output of translation. Since then, the mainstream keyword generation methods became based on Sequence-to-Sequence model (Seq2Seq) [4] such as what Meng et al. [6] introduced in a model based on CopyRNN to generate keywords in academic texts. They took the generation process as a Sequence-to-Sequence learning task framework, and employed a widely used encoder-decoder framework with attention and copy mechanisms. Chen et al. [7] proposed CorrRNN model to capture the correlation between multiple keywords. However, these Recurrent Neural Network (RNN) based models may suffer the low-efficiency issues. Because of the computation dependency between the current time step and the preceding time steps in RNN [5], Zhang et al. [8] proposed CopyCNN model based on convolutional neural network (CNN). It employs position embedding for obtaining a sense of order in the input sequence and adopts Gated Linear Units (GLU) as the nonlinearity function. In addition, some extraction methods also considered the influence of title, such as that Li et al. [16] introduced a graph-based ranking algorithm which sets the importance of words in the title to one and the others as zero, then propagates the influence of title phrases iteratively.

### 2.2. Topic Modeling

Keywords can represent the topics of a document. A document is usually composed of multiple semantic topics. Therefore, the extracted keywords should also cover all topics in the document. Li et al. [17] proposed the single topical PageRank (single TPR) method to calculate the probability of words under all topics of the document without decomposing into multiple PageRank models, which greatly reduces the amount of calculation. Parveen et al. [18] proposed the salience rank model to balance the topic specificity and corpus specificity of words and avoid extracting words that are not highly related to the topic. Our work is closely related to topic models. Topic-aware is to use topic model to find latent topics from document level word co-occurrence, and then join the model with keywords generation model. Starting from latent semantic analysis (LSA [19]), topic model is used to reveal the underlying semantic structure of document collection has been widely used in data mining, text processing, and information retrieval [3]. Among them, the typical topic models are probabilistic topic models (such as PLSA [20], LDA [21], and HDPs [22]). They provide an extensible basis for document modeling by referencing the latent topic of each variable in topic allocation [22]. With the wide application of deep learning technology in the field of natural language processing, some researchers have proposed a topic model based on neural network. This kind of method mainly uses neural network to reconstruct the text generation process of topic model and adds the sparse constraint of topic in the modeling to generate more expressive topic words [23]. We use a topic model based on variational autoencoder [24, 25] to infer latent topics, which is also conducive to the use of other neural models for end-to-end training without the need for specified model derivation. This model has been proved useful for citation recommendation [26] and conversation understanding [27]. Zeng et al. [28] proposed joint training topic model and short text classification model, but due to the diversity of keywords, this method cannot adapt to the scene of this work. Thus, this paper uses the neural topic model based on variational autoencoder to find the latent topics, which will also be trained together with the keyword generation model.

Sequence to sequence (seq2seq) model is a deep learning framework based on encoder and decoder. In 2014, Cho et al. [29] proposed seq2seq model based on cyclic neural network. This model uses the encoder and decoder to calculate the conditional probability of phrase pairs, which can improve the performance of machine translation. The Seq2seq can solve the problem of end-to-end sequence inequality and is suitable for a variety of natural language processing tasks. Using this model to generate keywords can generate keywords that have not appeared in the original document, which makes up for the shortcomings of the traditional keyword extraction model. The attention mechanism is also used in the coding process of this method, but it treats the title and the text alike.

## 3. Our Proposed Model

### 3.1. The Framework of KGM-TT

The traditional keyword extraction method cannot obtain the words that do not appear in the document. The existing generative methods ignore the guiding effect of document title on keywords and do not consider the subject semantic information of the document. The KGM-TT is a keyword generation model based on the fusion of topic aware and title guide, including neural topic model, title-guide hierarchical encoder, and topic-aware sequence decoder. The proposed KGM-TT integrates the semantic guidance of title words into the matching layer in the coding stage. The specific method is to use the attention mechanism to aggregate the title information for each word in the document content (Title-guide). In addition, in the decoding process, using the results of the trained neural topic model, a decoder with topic aware ability is improved to generate keywords with topic sensitivity (Topic-aware).

The framework of KGM-TT model is shown in Figure 2. First, the corpus is preprocessed, and the document topic distribution is generated by neural topic model. Then, the corpus is encoded by the title-guide hierarchical encoder. Finally, the topic distribution and coding representation are input into the topic aware sequence decoder to decode and automatically generate keywords. The training process of the left neural topic model in the framework is used to obtain the topic distribution of the document. The right branch of the frame is the encoding process of the document word sequence. Different from reference [29], we use the title to guide the word coding in the document in the coding stage. In addition, in the decoding stage, the topic of document in the right branch is integrated. The measures of Title-guide and Topic-aware make our KGM-TT better than other models, such as references [6, 8, 9].

### 3.2. Neural Topic Model

The neural topic model (NVDM-GSM) is used in KGM-TT is based on variational autoencoder (VAE). As shown in Figure 3, it is composed of an encoder and a decoder to simulate the process of document reconstruction [24].

Specifically, the document *C*={*X*_1_, *X*_2_, ⋯, *X*_*L*_} in corpus *C* as input, and process each document *X* into a BoW vector *X*_bow_. *X*_bow_ is the *V*-dimensional vector on the vocabulary (*V* is the size of the vocabulary), input *X*_bow_ into the neural topic model and encode it into a continuous Gaussian variable *Z* (representing *X*'s topic) by BoW encoder. Then the BoW decoder with *Z* as the condition reconstructs *X* and outputs a BoW vector *X*_bow_′. The decoder simulates topic model's generation process. We then describe their division of labor.

*BoW Encoder*. Bow encoder is used to estimate a priori variables *μ* and *σ*, and *σ* is used to lead out topic representation *Z*. We adopt the following formula:

(1) $$\begin{array}{c} \mu =f_{\mu }\left(f_{e}\left(X_{\text{bow}}\right)\right),\text{ log}\sigma =f_{\sigma }\left(f_{e}\left(X_{\text{bow}}\right)\right). \end{array}$$

where *f*_*∗*_(·) is a neural perceptron with an RuLU activated function.

*BoW Decoder*. Suppose that the attributive database *C* has *K* topics, and the topic vocabulary distribution of each topic in the vocabulary is represented by *ϕ*_*K*_. For each document *X* ∈ *C*, there is a document subject distribution represented by *θ* (*K*-dimensional). Specific to the neural topic model, *θ* is constructed by *softmax* functions. The generation process of documents in the decoder is as follows:

1. Draw latent topic variable *Z* ~ *N*(*μ*, *σ*^2^)
2. Using softmax function construction topic mixture *θ*=softmax(*W*_*θ*_^*T*^*Z*)
3. For each word, *w* ∈ *X*, *w* ~ softmax(*W*_*ϕ*_^*T*^*θ*)

Here *N*(*μ*, *σ*^2^) represents the multidimensional Gaussian distribution, and *σ*^2^ is the diagonal of the covariance matrix. *W*_*θ*_ is the matrix of *L∗K*, *L* is the dimension of *Z*, and *K* is the number of topic. Here, it is used as the topic-word distributions (*ϕ*_1_, *ϕ*_2_, ⋯, *ϕ*_*K*_). We adopt the topic mixture vector *θ* as the topic representation to guide keyword generation.

### 3.3. Title-Guide Hierarchical Encoder

As shown in Figure 4, the title-guide hierarchical encoder module is composed of sequence encoding layer, matching layer, and merging layer. The sequence encoding layer reads the title input and main body input and learns their context representation, respectively. The matching layer matches the relevant title information for each word of the document, reflecting the important words in the document. The merging layer merges the aggregated title information into each word to generate a title-guide context representation.

#### 3.3.1. Sequence Encoding Layer

The vector table maps each word in the text and title to a dense vector with a fixed size *d*_*e*_. Two bidirectional Gate Recurrence Units (GRU) [29] are used to encode the context and title, respectively, and the context information is combined into the representation of each word. The specific formula is as follows:

(2) $$\begin{array}{c} {\overset{⟶}{u}}_{i}=GRU_{11}\left(x_{i},{\overset{⟶}{u}}_{i-1}\right),\\ {\overset{\leftarrow }{u}}_{i}=GRU_{12}\left(x_{i},{\overset{\leftarrow }{u}}_{i+1}\right),\\ {\overset{⟶}{v}}_{j}=GRU_{21}\left(t_{j},{\overset{⟶}{v}}_{j-1}\right),\\ {\overset{\leftarrow }{v}}_{j}=GRU_{22}\left(t_{j},{\overset{\leftarrow }{v}}_{j+1}\right),\\ u_{i}=\left[{\overset{⟶}{u}}_{i};{\overset{\leftarrow }{u}}_{i}\right],\\ v_{j}=\left[{\overset{⟶}{v}}_{j};{\overset{\leftarrow }{v}}_{j}\right], \end{array}$$

where *i*=1,2, ⋯, *L*_*x*_, *j*=1,2, ⋯, *L*_*t*_, *x*_*i*_ is the vector of the *i*-th word of the document in the corpus, *t*_*j*_ is the vector of the *j*-th word of the document title. *u*_*i*_ and *v*_*j*_ is the context vector of the *i*-th word and the *j*-th title word, ${\overset{⟶}{u}}_{i},{\overset{\leftarrow }{u}}_{i},{\overset{⟶}{v}}_{j},{\overset{\leftarrow }{v}}_{j}$ is the hidden vector of *d*/2 dimension, where *d* is the hidden layer dimension of bidirectional GRU. ⟶ indicates the coding direction to the right and ← indicates the coding direction to the left.

#### 3.3.2. Matching Layer

The attention-based matching layer is engaged to aggregate the relevant information from the title for each word within the context. The aggregation operation *c*_*i*_=attn(*u*_*i*_, [*v*_1_, *v*_2_, ⋯, *v*_*L*_*t*__]; *W*_1_) is as follows:

(3) $$\begin{array}{c} c_{i}=\sum_{j=1}^{L_{t}}\alpha_{i,j}v_{j},\\ \alpha_{i,j}=\frac{\exp\left(s_{i,j}\right)}{\sum_{k=1}^{L_{t}}\exp\left(s_{i,k}\right)},\\ s_{i,j}={\left(u_{i}\right)}^{T}W_{1}v_{j}. \end{array}$$

where *c*_*i*_ the aggregated information vector of the *i*-th word of document *x*, *s*_*i*,*j*_ is the unnormalized attention between *u*_*i*_ and *v*_*j*_, *α*_*i*,*j*_ is the normalized attention between *u*_*i*_ and *v*_*j*_.

Documents contain title and main body, so the matching layer is also composed of two parts. One part is title-to-title self-matching, in order to better contact the context information of each title word. Because the title contains a lot of high summary information, this part is used to strengthen the importance of the title itself and plays a vital role in capturing the important information of the document. The other part is the matching from main body to title. Each word in the text aggregates the information of the title according to semantic relevance. This part is used to highlight the words highly related to the title, and use the title information to reflect the importance of the words in the text. Compared with the previous Sequence-to-Sequence methods, this matching layer makes full use of the summary information contained in the title.

#### 3.3.3. Merging Layer

The source contextual vector *u*_*i*_ and the aggregated information vector *c*_*i*_ are used as the input to the information merging layer. The specific formula is as follows:

(4) $$\begin{array}{c} {\overset{⟶}{m}}_{i}=GRU_{31}\left(\left[u_{i};c_{i}\right],{\overset{⟶}{m}}_{i-1}\right),\\ {\overset{\leftarrow }{m}}_{i}=GRU_{32}\left(\left[u_{i};c_{i}\right],{\overset{\leftarrow }{m}}_{i+1}\right),\\ {\tilde{m}}_{i}=\lambda u_{i}+\left(1-\lambda \right)\left[{\overset{⟶}{m}}_{i},{\overset{\leftarrow }{m}}_{i}\right],\\ M=\left[{\tilde{m}}_{1},{\tilde{m}}_{2},\cdots ,{\tilde{m}}_{L_{x}}\right], \end{array}$$

where *u*_*i*_ is a residual connection, *λ* ∈ (0,1) is the corresponding hyperparameter. Finally, the title-guide context representation $\left[{\tilde{m}}_{1},{\tilde{m}}_{2},\cdots ,{\tilde{m}}_{L_{x}}\right]$ is obtained and stored as *M* for subsequent decoding process.

### 3.4. Topic-Aware Sequence Decoder

As shown in Figure 5, the topic aware sequence decoder is conditional on encoding representation *M* and latent topic *θ*, the generation process of the following keyword *Y* is defined:

(5) $$\begin{array}{c} \text{Pr}\left(Y|X\right)=\prod_{j=1}^{\left|y\right|}\mathrm{Pr}\left(y_{i}|Y_{\langle )j},M,\theta \right). \end{array}$$

where *Y*_〈*j*_=〈*y*_1_, *y*_2_, ⋯, *y*_*j*−1_〉, Pr(*y*_*j*_*|Y*_〈*j*_, *M*, *θ*), denoted as *p*_*j*_, is a word distribution over vocabulary, reflecting how likely a word to fill in the *j*-th slot in target keyword.

The sequence decoder adopts a unidirectional GRU. On the general state update, the *j*-th hidden state *s*_*j*_ is further designed to add the latent topic *θ* of the document *X*:

(6) $$\begin{array}{c} s_{j}=f_{GRU}\left(\left[z_{j};\theta \right],s_{j-1}\right), \end{array}$$

where *z*_*j*_ is the input of the *j*-th decoder, *s*_*j*_ is the hidden state at the *j*-th time, *s*_*j*−1_ is the previous hidden state, and [; ] indicates the connection operation.

The decoder decodes sequence *M* and obtains key information through the attention mechanism. When predicting the *j*-th word in the keyword, the attention weight on *w*_*i*_ ∈ *X*_*seq*_ is defined as *α*_*ij*_′:

(7) $$\begin{array}{c} \alpha_{ij}^{'}=\frac{\exp\left(f_{\alpha }\left({\tilde{m}}_{i},s_{j},\theta \right)\right)}{\sum_{i\prime }^{\left|X\right|}\exp\left(f_{\alpha }\left({\tilde{m}}_{i\prime },s_{j},\theta \right)\right)},\\ f_{\alpha }\left({\tilde{m}}_{i},s_{j},\theta \right)=v_{\alpha }^{T}\tanh\left(W_{\alpha }\left[{\tilde{m}}_{i};s_{j};\theta \right]+b_{\alpha }\right), \end{array}$$

where *v*_*α*_, *W*_*α*_, *b*_*α*_ are trainable parameters and *f*_*α*_(·) indicates the semantic relationship between the *i*-th word and the *j*-th target word to be predicted. This relationship is also calibrated with the input latent topic information *θ* to explore and highlight the topic words. Thus, the topic sensitive context vector *c*_*j*_ is obtained:

(8) $$\begin{array}{c} c_{j}=\sum_{i=1}^{\left|X\right|}\alpha_{ij}^{'}{\tilde{m}}_{i}. \end{array}$$

In addition, under the condition of *c*_*j*_, the *j* th word is generated on the vocabulary according to the following formula:

(9) $$\begin{array}{c} p_{\text{gen}}=\text{softmax}\left(W_{\text{gen}}\left[s_{j};c_{j}\right]+b_{\text{gen}}\right). \end{array}$$

A copy mechanism See et al. [30] is added here to extract keywords from the source document. Specifically, *λ*_*j*_ ∈ [0,1] is used as a soft switch to decide whether to copy a word directly from the original text as the *j*-th target word.

(10) $$\begin{array}{c} \lambda_{j}=\text{sigmoid}\left(W_{\lambda }\left[z_{j};s_{j};c_{j};\theta \right]+b_{\lambda }\right), \end{array}$$

where *W*_*λ*_, *b*_*λ*_ are trainable parameters and topic information *θ* is also injected here to guide the switch decision.

Finally, the distribution *p*_*j*_ of the *j*-th target word can be predicted by using the following formula:

(11) $$\begin{array}{c} p_{j}=\lambda_{j}\cdot p_{\text{gen}}+\left(1-p_{\text{gen}}\right)\cdot \sum_{i=1}^{\left|X\right|}\alpha_{ij}^{'}, \end{array}$$

where attention scores {*α*_*ij*_′}_*i*=1_^|*X*|^ serve as the extractive distribution over the source input.

### 3.5. Jointly Learning Topics and Keywords

Our model KGM-TT is an end-to-end learning of latent topic model and keyword generation. First, the objective functions of the two modules are defined, respectively.

For the neural topic model, the objective function is defined based on negative lower bound of negative variation, and its loss function is as follows:

(12) $$\begin{array}{c} L_{GSM}=D_{KL}\left(p\left(Z\right)\left\|\right)q\left(Z|X\right)\right)-{Ε}_{q\left(Z|X\right)}\left[p\left(X|Z\right)\right]. \end{array}$$

where the first term is the Kullback–Leibler divergence loss and the second term reflects the reconstruction loss. *p*(*Z*) represents a priori distribution, *q*(*Z|X*) and *p*(*X|Z*) represent the process of BoW encoder and BoW decoder, respectively.

For the keyword generation model, the minimum cross entropy loss function is used for training on all training sets:

(13) $$\begin{array}{c} L_{KG}=-\sum_{n=1}^{N}\log\left(\mathrm{Pr}\left(Y_{n}|X_{n},\theta_{n}\right)\right), \end{array}$$

where *N* is the number of instances of the training set and *θ*_*n*_ is *X*_*n*_ 's latent topics induced from GSM.

Finally, the linear combination of *L*_*GSM*_ and *L*_*KG*_ is used to define the training objectives of the whole framework:

(14) $$\begin{array}{c} L_{KG-CTATG}=L_{GSM}+L_{KG}, \end{array}$$

where *γ* hyperparameters balance the effects of neural topic model and generative model.

The two models are trained together and their parameters are updated at the same time. After the training, the beam search is used to generate the ranking list of keywords.

## 4. Experiment and Analysis

### 4.1. Experimental Data

The corpus CNKI is crawled by our own crawler from China's largest scientific and technological publications databases (https://www.cnki.net). It has 18,000 papers in total and includes 5,6589 words. These documents are papers published from 2000 to 2020, including the title, abstract content, keywords, and publication time of the paper. In order to reflect its good portability and achieve good results in large-scale data sets, the largest publicly available keyword generation data set KP20k built by Meng et al. [8] in 2017 is selected for testing and evaluation in our experiment. The KP20k consists of a large number of high-quality scientific publications from different fields of computer science. The details of CNKI and KP20k are shown in Table 1.

### 4.2. Parameter Setting

For the neural topic model, it is implemented according to the design of Zeng et al. [28] and the number of topics *K* is set to 50. For the hierarchical encoder, the vocabulary *V* is defined as 50,000 words with the highest frequency of use. Set the embedding dimension *d*_*e*_ to 100, the number of hidden nodes to 256, the damping coefficient *λ* to 0.5, and the word embedding is randomly initialized and evenly distributed in [−0.1, 0.1]. Using the optimization model of Adam et al. [31], the batch size is 64, the initial learning rate is set to 10^−4^, the gradient cutting is set to 1, and the launch rate is set to 0.1. The convergence speed of neural topic model is much slower than that of generative model. Therefore, before joint training, train the neural topic model for 100 iterations and the generative model for 1 iteration. Empirically set *γ* = 1.0 to balance the loss of neural subject model and generation model, and iteratively update the parameters in each module. Then update their combination in turn. In the test, set the maximum depth of beam search to 6 and the beam size to 200.

### 4.3. Evaluating Indicator

We use Precision (P) to measure the accuracy of the model, Recall (*R*) to measure the integrity of the model, and *F*1-measure to evaluate the performance of keyword extraction methods. *T*_*o*_ represents the keyword set provided by the dataset itself, *T*_*e*_ represents the keyword set extracted by the model, and *T*_*o*_∩*T*_*e*_ represents the correctly extracted keyword set. Precision, Recall, and *F*1-measure are defined as follows:

(15) $$\begin{array}{c} p=\frac{\left|T_{o}\cap T_{e}\right|}{\left|T_{o}\right|},\\ R=\frac{\left|T_{o}\cap T_{e}\right|}{\left|T_{e}\right|},\\ F1-\text{Measure}=\frac{2\times P\times R}{P+R}. \end{array}$$

### 4.4. Experimental Results and Analysis

For the keyword prediction existing in the source text, two unsupervised models, including TF-IDF and TextRank, and a supervised model KEA are used as the traditional extraction method. In addition, the following keyword generation models are considered: Sequence-to-Sequence (Seq2Seq) model without copy mechanism, sequence-to-sequence model with copy mechanism CopyRNN and CopyCNN. For the prediction of keywords that do not exist in the source text, since the traditional extraction methods cannot generate such keywords, the baseline models are CopyRNN and CopyCNN. For all baseline models, select the same parameter settings as Meng et al. [6].

For predicting the keywords existing in the source text, the keyword prediction ability of the above model on CNKI and KP20k datasets is compared. The *F*1-measure values of the top 5 and top 10 predictions of each model are shown in Table 2.

It can be found from the table that all the generation models are better than the traditional baseline method. In addition, it can be noted that the model proposed in this paper has significant advantages in both datasets. For example, on the KP20k dataset, our model improves 15.2% (*F*1@10 score) than the best generative model CopyCNN. Generally speaking, the recall rate (*R*) of the top 10 and top 50 predictions is engaged as an indicator to measure how many absent keywords are correctly predicted. The experimental results are shown in Figure 6.

On the two datasets, we observed that our model is always better than the previous sequence to sequence model, such as our model is on the kp20k dataset, R@10 score is 10.2% higher than CopyCNN model. In general, the results show that our model can generate keywords better than the baseline model and capture the latent semantic information in the context content.

The quality judgment of keywords is controversial. Therefore, in addition to the above objective evaluations, we also invited five artificial experts to evaluate the prediction results of the models. Each expert was given the task of judging 100 papers. They need to judge the right and wrong results of the three generative keyword models: CopyRNN, CopyCNN, and our KGM-TT. For fairness, hide the models name in the expert evaluation process. We conducted the experiment on Chinese corpus CNKI and selected five keywords for evaluation. The experimental results are shown in Table 3.

According to the judgment results of artificial experts in Table 3, the *F*1 index of model CopyRNN and model CopyCNN is basically close. In contrast, the KGM-TT is ahead, about 5 percentage points higher than the other two models. The specific reason is the KGM-TT use the attention mechanism to aggregate the title information for each word in the document content and use a decoder with topic aware ability. It is improved to generate keywords with topic sensitivity.

## 5. Conclusion

The traditional keyword extraction method and cannot obtain the words that do not appear in the document. The existing generative methods ignore the guiding effect of document title on keywords and do not consider the subject semantic information of the document. We present a keyword generation model based on combination topic aware and title-guide (KGM-TT). In the process of encoding document words, it is guided by the title semantics. In the decoding process, a topic aware decoder is used. Therefore, the keywords generated by the KGM-TT are more subject-sensitive and higher quality. The experimental results show that the KGM-TT model proposed in this paper can make better use of the strong semantic information of the latent topic and title of the document. The KGM-TT is superior to other methods in keyword prediction, and can generate keywords with high accuracy. However, there are a large number of synonyms in the words generated by the keyword generation model. This is a problem that needs to be solved in our research in the future.

## Figures and Tables

**Figure 1:** An example of keyword generation.

**Figure 2:** KGM-TT framework.

**Figure 3:** Neural topic model.

**Figure 4:** The title-guide hierarchical encoder module.

**Figure 5:** The title-guide hierarchical decoder module.

**Figure 6:** Absent keyword predicting results.

**Table 1:** The number of experimental documents and its division.

Corpus	Training	Verification	Verification	Total
CNKI	12,600	3,600	1,800	1,8000
KP20k	530,809	20,000	20,000	570,809

**Table 2:** Present keyword predicting results.

	Model	CNKI		KP20k	
		F1@5	F1@10	F1@5	F1@10
Extractive models	TF-IDF	0.233	0.311	0.104	0.126
	TextRank	0.324	0.302	0.176	0.147
	KEA	0.336	0.328	0.180	0.163
Generative models	Seq2Seq	0.417	0.392	0.243	0.216
	CopyRNN	0.486	0.424	0.321	0.260
	CopyCNN	0.518	0.473	0.349	0.283
	KGM-TT	0.602	0.569	0.392	0.334

**Table 3:** Expert evaluation results.

	CopyRNN	CopyCNN	KGM-TT
F1@5	0.529	0.531	0.587

## Data Availability

The data generated and analyzed during this research are available from the corresponding author on request.
